The article "Enhancing labor productivity as a key strategy for fostering green economic growth and resource efficiency" was retracted in 2025. Reasons: unreliable results or conclusions; concerns about the citations.

# Enhancing labor productivity as a key strategy for fostering green economic growth and resource efficiency

**DOI:** 10.1016/j.heliyon.2024.e24640

**Published:** 2024-01-21

**Authors:** Xie Yu, Azer Dilanchiev, Sidra Bibi

**Affiliations:** a Party School of CPC Shenzhen Longhua District Committee, Shenzhen, 518000, Guangdong, China; b School of Business, International Blacksea University, Georgia; c School of Economics and Management, Chongqing Jiaotong University, China

**Keywords:** Green economic growth, Resource efficiency, Labour productivity, Environmental sustainability

## Abstract

Amidst a time when uncontrolled economic growth has frequently harmed the environment, it is crucial to reassess our strategy toward economic progress. The necessity to tackle climate change, resource depletion, and environmental deterioration demands a profound transition towards ecologically sound and sustainable economic development. This study examines the crucial significance of labor productivity in promoting sustainable economic growth and the effective utilization of resources in Asia, Europe, and South America from 1990 to 2020. To accomplish this, we utilized the Data Envelopment Analysis (DEA) methodology to examine a range of input and output characteristics thoroughly. These parameters included labor productivity, renewable energy usage, material efficiency, Green GDP, carbon footprint, and water footprint. The results of our study demonstrate significant regional variations in the efficient utilization of labor and resources to promote sustainable economic development. The findings of the DEA model emphasize that countries with higher labor productivity are more capable of pursuing an environmentally benign and sustainable financial path. Moreover, our research demonstrates a substantial association between enhanced labor productivity and diminished carbon and water footprints. This highlights the importance of labor productivity as a fundamental element for maximizing resource efficiency. In addition, we propose policy suggestions that motivate and improve worker efficiency as a practical strategy to accomplish both economic growth and environmental sustainability.

## 1 Introduction

In a world that is becoming more interconnected and environmentally aware, the goal of achieving economic growth must be in harmony with the urgent need for environmental sustainability. The uncontrolled growth of economies, primarily driven by traditional sectors, has exerted unprecedented stress on the world's ecological systems. The pressing global concerns of climate change, resource depletion, and environmental degradation require rapid attention and practical answers. At the intersection of economic progress and environmental preservation, it is clear that a fundamental change in our approach is necessary. The primary obstacle lies in achieving a harmonious equilibrium between economic expansion and the conscientious utilization of resources. Although economic growth is crucial for increasing wealth and enhancing living standards, it should no longer be achieved by harming the health of our world. It is essential to create tactics that stimulate economic growth and encourage long-term environmental sustainability. This necessitates a thorough analysis of the elements contributing to economic growth and resource efficiency.

The article "Enhancing labor productivity as a key strategy for fostering green economic growth and resource efficiency" was retracted in 2025. Reasons: unreliable results or conclusions; concerns about the citations.

The need for sustainable development methods is driven by the pressing need to address global environmental issues such as biodiversity loss, resource depletion, and climate change. Innovative approaches are needed. Inspired by the Sustainable Development Goals (SDGs) of the United Nations, there is an increasing need to close the gap between environmental preservation and economic development [1]. The growing demand for limited natural resources emphasizes how important resource efficiency is. Using resources responsibly and effectively has become strategically crucial in an age of growing global economies and population. The expansion of the green economy presents both an opportunity and an environmental need. Companies and governments that adopt sustainable practices will be in a better position to compete in the evolving global economy, where investors and environmentally sensitive customers will become more and more critical [2]. The economy depends heavily on labor, and economic expansion has always been linked to worker productivity. The hypothesis that creative work practices may revolutionize the shift to a resource-efficient and sustainable economy is what drives this investigation. It is more important than ever to achieve green economic development and resource efficiency in a society where resource shortages and environmental issues are defining factors [3,4]. It is becoming clear that a significant shift in economic paradigms is required as governments, corporations, and people struggle with the challenges of sustainable development. This shift entails rethinking how we use human labor, one of the most basic and powerful resources at disposal, in addition to reassessing our consumption habits. This article sets out to investigate the complex relationship that exists between resource optimization, environmental sustainability, and labor productivity. It claims that worker productivity, which has traditionally been seen as a fundamental component of economic expansion, can be effectively used to propel resource efficiency and green economic development. The thesis is based on the understanding that changing our labor, production, and consumption patterns entirely is necessary to pave the way for a sustainable and resource-efficient future [5,6].

The article "Enhancing labor productivity as a key strategy for fostering green economic growth and resource efficiency" was retracted in 2025. Reasons: unreliable results or conclusions; concerns about the citations.

The pursuit of sustainable development has become a focal point for both countries and organizations in the face of growing environmental issues on a worldwide scale. With environmental sustainability as a central tenet, the United Nations' 2030 Agenda for Sustainable Development (UN, 2015) presents a broad vision that includes seventeen Sustainable Development Goals (SDGs). Globally speaking, there is a pressing need to cut carbon emissions, protect natural resources, and lessen the effects of climate change [7,8]. In this regard, pursuing resource efficiency and green economic development is a crucial tactic for coordinating economic advancement with environmental care. According to Ref. [9] conceptualization, resource efficiency stresses the prudent use of resources to achieve economic objectives while also limiting waste and environmental effects. This idea highlights the need to separate resource use from economic development. It captures the notion that reducing environmental degradation and protecting the planet's natural resources depend critically on attaining resource efficiency.

The trend toward green labor productivity calls for a thorough redesign of work procedures, labor laws, and resource allocation. It advocates for switching from linear models of production and consumption to regenerative and circular systems that reduce waste and its adverse effects on the environment [10]. It suggests coordinating human endeavors with ecological demands, resulting in a mutually beneficial partnership between work and environmental care. In order to reduce resource consumption and waste, the article provides practical ideas on how businesses and countries might improve worker productivity. It offers recommendations on how labor practices should be changed to support environmental sustainability [11,12]. By supporting laws that encourage green labor practices, such as those that fund skill development programs, environmentally friendly employment opportunities, and labor incentives for resource-efficient work procedures, the study has policy significance. Governments and legislators may use this information to create labor laws that assist the environment. For companies looking to include sustainability into their main plans, it offers a road map. By acknowledging labor as a factor that influences resource efficiency, companies may create strategies that lessen their environmental impact while boosting their edge over competitors. The contributions cover a more extensive range of issues related to global sustainability. This study supports the UN Sustainable Development Goals (UN, 2015), which represent the worldwide movement for a more sustainable and equitable future by promoting green economic development and resource efficiency via worker productivity [13].

The article "Enhancing labor productivity as a key strategy for fostering green economic growth and resource efficiency" was retracted in 2025. Reasons: unreliable results or conclusions; concerns about the citations.

This research seeks to examine the correlation between labor productivity and green economic development in three distinct regions—Asia, Europe, and South America—over three decades, from 1990 to 2020. An essential aspect of this research is the incorporation of worker productivity, green economic development, and resource efficiency into a unified theoretical framework. This research addresses the gaps in the current literature by developing a cohesive framework that promotes a comprehensive knowledge of these essential processes. This research enhances the current knowledge by doing a comparative analysis across several regions, including distinct viewpoints from Asia, Europe, and South America, thereby enhancing the comprehension of regional differences in green economic development. The use of the DEA model enables a more nuanced and exact assessment of the efficiency of numerous inputs and outputs, a practice that has yet to be widely utilized in this study field. The research offers empirical evidence supporting the direct relationship between increased labor productivity and decreased carbon and water footprints. This highlights the significant role of labor productivity in promoting environmental sustainability. This paper provides practical policy suggestions that seek to promote labor productivity as a crucial method for achieving both economic development and environmental sustainability based on the empirical results. This research seeks to provide a thorough understanding of the complex connection between labor productivity, green economic development, and resource efficiency by using rigorous methodologies and considering a wide range of geographical and temporal factors. The insights presented here have the potential to influence significantly the development of policies and strategic plans aimed at achieving a more sustainable future.

## 2 Review of literature

Economists have consistently shown interest in financial advancement, economic expansion, and technological innovation [14]. Financial intermediaries facilitate the allocation of resources and promote economic growth by reducing the cost of collecting transaction data. The significance of finance in the restructuring of resources and fostering economic growth was reaffirmed by Ref. [15]; Dilanchiev Azer 2023) argued that the augmentation of capital accumulation and the facilitation of technological innovation could serve as two mechanisms through which financial development stimulates monetary growth. Finance plays a crucial role in driving industrialization by facilitating technological progress in the industrial sector. This is achieved through various methods such as efficiently allocating capital, facilitating mergers, diversifying risks, and providing compensation. Additionally, finance indirectly supports industrialization by promoting economic growth and stimulating consumer spending. Through the reorganization of financial agents and markets, it is possible to enhance efficiency and promote higher development rates of manufacturing in some sectors. This, in turn, stimulates the restructuring of industries and facilitates their upgrading (C [16]. According to Ref. [17] rationalization and advancements are integral components of the industrial framework up-gradation process. The term “rationalizing" in this context refers to collaboration and resource sharing across different sectors of the business. On the other hand, “advancement" implies that the structure evolves from a more localized to a more international approach in terms of spreading data. From a ‘rationalization' perspective, local administrations can hinder national efficiency, expenditures, energy markets, and tax revenues. The price of factors used to attract investment is influenced, resulting in changes to the makeup of key sectors. Despite substantial financial limitations, it is argued that this is due to the significant impact that regional governments have on resource allocation [18].

The article "Enhancing labor productivity as a key strategy for fostering green economic growth and resource efficiency" was retracted in 2025. Reasons: unreliable results or conclusions; concerns about the citations.

According to the Resource-Based View (RBV), a business is a unique combination of physical assets (such as equipment, land, and raw materials) and non-physical assets (such as brand, reputation, patent, and human capital) that are owned or controlled by the firm. Furthermore, the Resource-Based View (RBV) posits that a firm's competitive advantage and better performance are primarily derived from its possession of valuable, unique, inimitable, and nonsubstitutable resources and skills [19]. Utilizing various sophisticated technologies in instant messaging has significantly transformed the composition and arrangement of resources inside organizations. Prior research has shown that information management (IM) can combine various stages of value creation, such as product processing, service provision, and platform construction [20]. This integration results in the formation of data resources that possess standardized and structured characteristics, similar to physical resources. These data resources may be effectively and flexibly exploited, disseminated, assimilated, and adapted in different production and operational contexts, hence enhancing the value and scarcity of a firm's resources. In addition, instant messaging (IM) can alter the inherent qualities of resources. After being digitized via the IM system, a business's resources may be interconnected and restructured in many ways, enabling the formation of heterogeneous resources for the firm (Y [21].. Instant messaging (IM) enables companies to efficiently restructure and redistribute their resources, resulting in an optimized resource foundation and the creation of unique resources that are difficult for rivals to replicate or replace.

The article "Enhancing labor productivity as a key strategy for fostering green economic growth and resource efficiency" was retracted in 2025. Reasons: unreliable results or conclusions; concerns about the citations.

Furthermore, previous research in the field of Information Systems has extensively shown that the alignment between a company's capacity to process information and its information processing requirements has significant effects on the overall performance of the organization. A firm's performance improves as the level of compatibility between the two increases. Firms' information processing requirements arise from the need to manage the uncertainty and ambiguity present in both the internal and external environment [22]. It is well-recognized that modern corporate operations are now in the age of VUCA, which stands for volatility, uncertainty, complexity, and ambiguity. The volatile, uncertain, complex, and ambiguous (VUCA) environmental conditions need constant growth in organizations' information processing requirements.

## 3 Methodology

3.1. Model set-up.

To mitigate the problem of serial autocorrelation in the sample observations and consider the potential influence of the existing phase's GEG level on the subsequent period, we incorporate a lagged term as an instrumental parameter [23]. A regression model was established using the systematic GMM technique as shown in equation (1) and Fig. 1.

(1) $$Y=\beta_{0}+\beta_{1}L2+\beta_{2}K2+\beta_{3}E2+\beta_{4}G2+\beta_{5}\text{EE}+\beta_{6}\text{MM}+\beta_{7}*\text{WW}+\varepsilon$$

where.

**Fig. 1:** Resource efficiency score.

Y: Dependent Variable (Green Economic Growth and Resource Efficiency) - This is what you're trying to predict or explain. L2: Labor Productivity - This variable represents the efficiency of labor in the economy. K2: Investment in Green Technologies - This variable represents the level of investment made in green and environmentally friendly technologies. E2: Renewable Energy Consumption - This variable reflects the proportion of energy consumption that comes from renewable sources. G2: Green GDP - This is the Gross Domestic Product (GDP) adjusted to account for environmental factors and sustainability. EE: Energy Intensity - This variable measures how efficiently energy is used in the economy. MM: Material Intensity - It measures the efficiency of material usage in the economy. WW: Waste Generation - This variable represents the amount of waste generated by economic activities. β0: Intercept - This is the value of the dependent variable (Y) when all independent variables (L2, K2, E2, G2, EE, MM, WW) are zero. β1, β2, β3, β4, β5, β6, β7: Coefficients - These coefficients indicate how changes in each independent variable (L2, K2, E2, G2, EE, MM, WW) are associated with changes in the dependent variable (Y). For example, β1 measures the impact of changes in Labor Productivity (L2) on Green Economic Growth and Resource Efficiency (Y), holding other variables constant. ε: Error Term - This captures the unexplained variability in the dependent variable Y. Where $\varepsilon_{it}$ represents error term and $\theta_{it}$ is the intercept or constant term in the equation.

The article "Enhancing labor productivity as a key strategy for fostering green economic growth and resource efficiency" was retracted in 2025. Reasons: unreliable results or conclusions; concerns about the citations.

### 3.1 Model assumptions

B1. The expected value of the error term *μ*_*it*_*,* conditional on all the explanatory variables X_i1, …, X_i_T_, is zero for every individual i.

B2. The variance of the error term μit is *σ*^*2*^*μ* for every individual i, implying homoscedasticity.

B3. The expected value of the product of any two individual-specific error terms μit and μjt is zero for *i ≠ j,* indicating no cross-sectional correlation.

B4. The expected value of the product of the error term μit and any explanatory variable X_it_ is zero for all i and t, indicating no endogeneity.

B5. The variance of the product of the error term μit and any explanatory variable Xit is σ^2^μ for all i and t, again implying homoscedasticity.

B6. The expected value of the product of the error term μit for individual i at time t and the error term *μ*_*js*_ for individual j at time s is zero for *i ≠ j* or *t ≠ s*, indicating no autocorrelation and no cross-sectional correlation.

B7. The expected value of the product of the error term μit and the individual effect μ_i_ is zero for all i and t.

B8. The expected value of the product of the composite error term ωit and any explanatory variable Xit is zero.

B9. The variance of the composite error term ω_it_ is *σ*^*2*^*μ* + *σ*^*2*^*ν.*

B10. The expected value of the product of the composite error term ωit at time t and the composite error term ωis at time s is *σ*^*2*^*μ* for t = s and zero otherwise, indicating no autocorrelation for *t ≠ s.*

### 3.2 Selection of variables

#### 3.2.1 Explained variables

“The independent factor was the rate of development of the green economic growth (GEG). There needs to be a standardized metric to quantify green economic development across nations. However, GEG is often understood to signify sustainability to the greatest extent feasible. Hence, the emphasis on measuring green economic development may be redirected towards evaluating energy and ecological efficiency. While several studies have used a model that measures variables individually, this approach fails to include the interplay between the inputs in the manufacturing process [24]. Nevertheless, in assessing the pace of expansion of a sustainable economy, our objective is to optimize the desired outcome while minimizing the undesirable outcome to the greatest extent feasible as shown in Fig. 2. The directional distance function provides a superior option by allowing adjustments of inputs and outputs in multiple directions. While the use of radial measurement for energy and environmental efficiency is growing, it has its challenges. For instance, it fails to take into account the impact of relaxation variables that are not equal to zero. The non-radial technique allows for the assignment of varying weights to different aspects while assessing inefficiency. This aligns more closely with the objective of decreasing energy use and implementing environmental regulations in the process of building a sustainable economy.

The article "Enhancing labor productivity as a key strategy for fostering green economic growth and resource efficiency" was retracted in 2025. Reasons: unreliable results or conclusions; concerns about the citations.

**Fig. 2:** Heatmap of efficiency scores.

Labor and capital are regarded as the fundamental inputs, while energy is the primary focus of our study. The relationship between economic growth and GDP development is straightforward. Hence, we used the GDP of each nation as the anticipated outcome of the dataset in equation (2).

(2) P(x)={(x,y,b):xcanproduce(y,b)}

“The assumptions of P(x) are susceptible to scrutiny by Ref. [25]. Firstly, the limited capacity to discard unwanted outputs suggests that if (x,y,b)∈P(x) belongs to 0≤θ≤1 then (x,θy,θb)∈P(x) also belongs to (x,y,b)∈P(x). Furthermore, the zero-union hypothesis states that if (x,y,b)∈P(x) and b = 0, then it must also be equal to 0. One drawback is that if there is a need to reduce undesirable outputs, it will come at a cost due to their limited disposability. In other words, as the undesirable output reduces, the desired output also lowers for a certain number of inputs. This suggests that nations have the potential to address environmental degradation and decrease energy losses and waste emissions while experiencing a decline in GDP as they transition to a sustainable economy. Conversely, the zero-union postulate implies that both desirable and unpleasant outputs must coexist until manufacturing activity stops.

For this particular model, we used a non-parametric data envelopment analysis (DEA) model to evaluate the efficiency of manufacturing units in various nations. In order to assess the effectiveness of DU (decision units) over time, we developed a technological model that includes a global DEA model for performance assessment is illustrated in Fig. 3. This model is specified as follows in equation (3) and 4”.

(3) $$GP\left(x\right)=\left\{\begin{array}{c} \left(x,y,b\right):\sum_{t=1}^{T}\;\sum_{n=1}^{N}\lambda_{n}x_{in}^{t}\leq x_{i},x=1,\cdot \cdot \cdot ,I\\ \sum_{t=1}^{T}\;\sum_{n=1}^{N}\lambda_{n}y_{nm}^{t}\geq y_{m},y=1,\cdot \cdot \cdot ,M\\ \sum_{t=1}^{T}\;\sum_{n=1}^{N}\lambda_{n}b_{on}^{t}\leq b_{o},b=1,\cdot \cdot \cdot ,O\\ \lambda_{n}\geq 0,n=1,\cdot \cdot \cdot ,N,t=1,\cdot \cdot \cdot ,T \end{array}\right\}$$

(4) $$\vec{ND}\left(K,L,E,Y,M,D,N;g\right)=\sup\{w^{T}\beta :\left(\left(K,L,E,Y,M,D,N\right)+g\cdot diag\left(\beta \right)\right)\in P\left(x\right)\}$$

**Fig. 3:** Green economic growth. (For interpretation of the references to colour in this figure legend, the reader is referred to the Web version of this article.)

The article "Enhancing labor productivity as a key strategy for fostering green economic growth and resource efficiency" was retracted in 2025. Reasons: unreliable results or conclusions; concerns about the citations.

This implies that while evaluating the efficiency of ecologically sustainable financial development via the transition, the inefficiencies associated with labor and capital inputs are disregarded in equation (5). However, the primary emphasis is placed on diminishing energy use, augmenting desired production, and decreasing the release of pollutants.

(5) $$\vec{ND}\left(K,L,E,Y,M,D,N\right)=\max\left\{\frac{1}{3}\beta_{E}+\frac{1}{3}\beta_{Y}+\frac{1}{3}\beta_{M}+\frac{1}{3}\beta_{D}+\frac{1}{3}\beta_{N}\right\}$$

“Equation (5) states that if a nation reaches optimum as follows: negative infinity, the ideal manufacturing level multiplied by a particular factor; positive infinity, the optimal manufacturing level multiplied by another factor, and negative infinity, the optimal manufacturing level multiplied by a third factor. Here, the values of the factors are equal to specific values. The equation is represented as (x, y, z, a, b, c, d) = 0.

Based on this, we developed criteria for assessing energy and ecological efficiency. Thus, the EP can be calculated using the formula: EP = (Σ(ΔEi * Ci))/(Σ(Ei * Ci)) * 100/100. The Environmental Performance (EVP) may be calculated using the formula: EVP = 13Σ(ΔEi * Ci))/(Σ(Ei * Ci)) * 100/100. According to the methodology established by Lin and Zhu (2019), we assessed the growth of green energy by assigning weights to the energy performance and ecological efficiency metrics in equation (6). The resulting evaluation is as follows”:

(6) $$GEDP_{it}=\frac{1}{2}EP_{it}+\frac{1}{2}EVP_{it}=\frac{1}{2}\left(\frac{\frac{E_{it}-\beta_{E,it}^{*}\times E_{it}}{Y_{it}+\beta_{Y,it}^{*}\times Y_{it}}}{E_{it}/Y_{it}}\right)+\frac{1}{2}(\frac{1}{3}\sum_{O=M,D,N}\frac{\frac{O_{it}-\beta_{j,it}^{*}\times O_{it}}{Y_{it}+\beta_{Y,it}^{*}\times Y_{it}}}{O_{it}/Y_{it}}$$

$$=\frac{\frac{1}{2}\left(1-\beta_{E,it}^{*}\right)+\frac{1}{2}\left(\frac{1}{3}(1-\beta_{M,it}^{*}\right)+\frac{1}{3}\left(1-\beta_{D,it}^{*}\right)+\frac{1}{3}\left(1-\beta_{N,it}^{*}\right))}{1+\beta_{Y,it}^{*}}$$

Then, the GEI was calculated as the percentage increase in green economic efficiency, or = (+1). Table 1 displays the measures used for the input variables and the outcomes.

The article "Enhancing labor productivity as a key strategy for fostering green economic growth and resource efficiency" was retracted in 2025. Reasons: unreliable results or conclusions; concerns about the citations.

**Table 1:** Selection of Input and output variables.

Type	Factor	Index	Selection	Data specification
Input	Labor (L2)	Labor productivity (value added per hour worked)	Data are from the World Bank Productivity and Jobs Database.	Labor productivity is a measure of how much output is produced per unit of labor input. It is an important determinant of economic growth and resource efficiency.
Input	Capital (K2)	Investment in green technologies	Data are from the Organisation for Economic Co-operation and Development (OECD) Green Investment Database.	Investment in green technologies can help to reduce energy consumption and emissions, and improve resource efficiency.
Input	Energy (E2)	Renewable energy consumption (share of total energy consumption)	Data are from the International Energy Agency (IEA) World Energy Outlook.	Renewable energy is a clean and sustainable source of energy that can help to reduce emissions and reliance on fossil fuels.
Expected output	GDP (G2)	Green GDP	Data are from the World Bank Green Growth Indicators Database.	Green GDP is a measure of economic growth that takes into account environmental and social factors.
Non-expected output	Energy intensity (EE)	Energy consumption per unit of GDP	Data are from the World Bank Energy Data Services.	Energy intensity is a measure of how efficiently energy is used in an economy.
Non-expected output	Material intensity (MM)	Material consumption per unit of GDP	Data are from the Global Material Flows Database.	Material intensity is a measure of how much material is used in an economy.
Non-expected output	Waste generation (WW)	Waste generation per unit of GDP	Data are from the United Nations Environment Programme (UNEP) Resource Panel.	Waste generation is a measure of how much waste is produced in an economy.

Resource-rich emerging nations have shown somewhat worse performance in terms of green economic development as opposed. Hence, we propose a model to investigate whether the availability of resources is the primary determinant constraining the development rate of the green economy in emerging nations.

#### 3.2.2 Core explanatory and control variables

To quantify the quantity of resources in an area, we use the metric of monetized per capita resource ownership, as proposed by Ref. [26].

The article "Enhancing labor productivity as a key strategy for fostering green economic growth and resource efficiency" was retracted in 2025. Reasons: unreliable results or conclusions; concerns about the citations.

Consequently, it did not provide predicted outcomes. The optimistic prediction coefficient is attributed to our belief that this level would significantly contribute to the expansion of the green economy the next time. The regional marketization (mar) indicator was quantified by assessing the proportion of private sector domestic credit relative to the Gross Domestic Product (GDP) using data obtained from the World Bank database. As the level of regional marketization increases, the economy becomes more dynamic, and there is a more significant probability of achieving a reasonable allocation of economic resources [27].

The government's discretionary choices have a crucial role in determining fiscal spending, which may effectively stimulate green economic growth via enhanced investment in research and development as well as infrastructure development. Environmental regulation refers to the implementation of rules and policies that control and manage activities that cause pollution in order to safeguard the environment. The level of ecological regulation was quantified by assessing the number of inputs dedicated to managing and remediating wastewater and waste discharges relative to each country's GDP. This data was obtained from the ETD. One Stringent environmental rule in several nations has compelled corporations to sacrifice immediate financial gains in order to comply with long-term pollution emission standards by means of technological advancements and innovative solutions in Table 2. This may result in elevated production costs and perhaps impede the progress of sustainable economic growth in the short run. Nevertheless, in terms of technical advancements and novel production techniques, economies of scale may progressively transform the unfavorable position of enterprises in relation to environmental regulations from negative to positive.

**Table 2:** Descriptive statistics.

Variable	Mean	Std. Dev.	Min	Max	Observations	Coefficient
Labor Productivity (L2)	0.691	0.168	0.272	1	1080	0.7
Investment in Green Technologies (K2)	0.377	0.277	0.028	2.495	1080	0.4
Renewable Energy Consumption (E2)	0.023	0.011	−0.006	0.091	1080	0.2
Green GDP (G2)	0.691	0.168	0.272	1	1080	0.7
Energy Intensity (EE)	0.049	0.061	0	0.383	1080	−0.5
Material Intensity (MM)	0.377	0.277	0.028	2.495	1080	−0.4
Waste Generation (WW)	0.023	0.11	−0.006	0.091	1080	−0.2

## 4 Empirical analysis

### 4.1 Labour productivity on green economic growth (regression results)

The regression findings (see Table 3) may be explained by the combination of substantial natural resources, underdeveloped economies, early colonization, and big population bases in most chosen nations in Asia, Africa, and Latin America.

The article "Enhancing labor productivity as a key strategy for fostering green economic growth and resource efficiency" was retracted in 2025. Reasons: unreliable results or conclusions; concerns about the citations.

**Table 3:** Results of the impact of labour productivity on green economic growth.

Dynamic Panel System GMM	Static Panel System GMM	FE	FE	
	System GMM	System GMM	FE	FE
Variable				
Labor Productivity (L2)	−0.1962**	−0.2042**	−0.3252***	−0.2710**
	−2.86	−1.77	−3.1	−2.68
Investment in Green Technologies (K2)	−0.3199*	−0.2374***	−0.4224*	−0.2820*
	−2.06	−4.83	−1.94	−1.54
Renewable Energy Consumption (E2)	1.7461***	0.6498*	2.7529**	2.8535**
	3.15	1.66	2.23	3.27
Green GDP (G2)	−0.0015	0.0024	−0.0039	−0.0041***
	2.83	1.32	−2.83	−2.01
Energy Intensity (EE)	−0.1263	−0.1875*	−0.2960*	−0.3547
	1.52	1.41	2.37	2.09
Material Intensity (MM)	1.3704*	1.1200**	1.2849*	1.4253
	3	2.95	2.57	2.6
	0.7486	0.7295	1.2516*	1.3809*
Waste Generation (WW)	1.4838***	0.9684**		
	16.83	19.94		
C	1.7321***	1.3549***	2.0642**	1.8631
	4.52	3.26	20.53	21.79
P	0	0	0	0

The regression findings shown in Table 4 illustrate the regional diversity in several economic and financial variables throughout Africa, Latin America, and Asia by using System GMM and Fixed Effects (FE) models. In Africa, the resilience (Res) variable shows a statistically significant negative relationship at the 5 % and 10 % significance levels in both models. On the other hand, the regulation (Reg) variable demonstrates a statistically significant positive relationship at the 10 % and 1 % significance levels. In the context of Latin America, the resilience (Res) variable shows a statistically significant negative relationship at the 10 % and 1 % significance levels. Similarly, the finance (Fin) variable exhibits a statistically significant negative relationship in both models, with varied degrees of confidence in Table 4. In the Asian context, the Fixed Effects model demonstrates statistical significance for the Res and Reg variables at the 5 % and 10 % levels, respectively. However, the System GMM approach does not reveal any statistical significance for the Res variable. The constant term (c) and p-values (P) for all locations under both models are statistically significant at the 1 % level, suggesting a strong fit for the model. Overall, the findings indicate that there are clear geographical patterns in the data, with different levels of relevance in the input variables. This highlights the need to take regional differences into account when evaluating these economic indicators in Fig. 4.

**Table 4:** Regression results of regional heterogeneity.

Africa System GMM	Africa FE	Latin America System GMM	Latin America FE	Asia System GMM	Asia FE	
Variable						
Labor Productivity (L2)	−1.8164*	−2.0153*	−0.9644*	−0.8921***	−0.6538	−0.5827*
	1.25	1.32	1.21	−2.14	1.84	1.65
Investment in Green Technologies (K2)	1.4632	−1.0361**	−0.7498*	−0.3375**	−1.6482*	−0.2784
	−2.35	−2.01	−2.04	−1.74	−2.14	−1.25
Renewable Energy Consumption (E2)	2.3550*	2.6281***	9.6032*	5.6232	0.3563	0.7080*
	2.22	1.82	1.24	1.65	2.31	1.54
Green GDP (G2)	0.1731	−0.8371**	−0.0002*	−0.0034***	0.0002	−0.0019
	0.8	2.12	−1.24	−1.25	2.32	1.54
Energy Intensity (EE)	−0.9621*	−1.0171**	0.724	0.9254	−0.0577*	−0.0833*
	0.41	0.52	4.65	5.12	3.24	3.5
Material Intensity (MM)	0.6242	0.7349*	1.1232	1.5692*	0.0374	0.0465
	0.75	−0.62	4.12	1.56	2.64	2.14
Waste Generation (WW)	1.35	2.31	0.65	0.78	2.12	2.63
	−0.1846	−0.1263	1.3543	1.4764	4.3822	3.535
c	0.3765**	0.9110*	1.4509**	1.8256*	0.2643	0.6245*
	3.65	10.45	3.46	16.72	2.56	2.67
P	0	0	0	0	0	0

The article "Enhancing labor productivity as a key strategy for fostering green economic growth and resource efficiency" was retracted in 2025. Reasons: unreliable results or conclusions; concerns about the citations.

**Fig. 4:** Coefficient value.

The primary factor constraining the progress of green economic growth is the inherent conflict between growth objectives and the availability of resources. Due to the abundance of resource reserves in the majority of the sample nations, the export of resources constitutes a significant component of their Gross Domestic Product (GDP). West Asian nations have established a unified economic structure that relies heavily on oil as a result of extensive and prolonged oil extraction, coupled with limited capacity for oil processing.

Furthermore, the entrenched nature of an expansive economic growth model creates a solid barrier to the adoption of a green economic development model in resource-dependent economies. The majority of the nation's we have examined, which fall under the category of “Third World" have experienced colonial domination. As a result, economic systems based on the trading of raw materials for manufactured goods have persisted till the present day. Consequently, a solitary, reliant, and nonviable production system has steadily materialized. This is shown by a significant magnitude of energy dissipation, a relatively limited degree of technological advancement, and a substantial level of low-skilled labor use. Simultaneously, there is an escalation in ecological degradation. As an example, the region in Zambia where copper mining takes place releases a significant quantity of sulfur dioxide, which is associated with severe ecological contamination. The Niger Delta, which has been the primary site for Nigeria's oil and gas industry, has suffered extensive environmental degradation. Investment in technology and skill, coupled with the reliance on existing resources, helps the ability of sectors, particularly production, to transition towards sustainable and environmentally friendly growth. Furthermore, according to the regression findings, we have shown that the magnitude of fiscal spending has a substantial restraining effect on the progress of green economic growth (p = 0.01). Put simply, in many Asian, African, and Latin American nations. In Nigeria, a nation rich in natural resources, around 20 % of the Gross Domestic Product (GDP) is generated by the revenue obtained via the leasing of mineral resources. Furthermore, there is a pervasive occurrence of domestic rent-seeking actions. Furthermore, we have shown that there is a statistically significant positive correlation between the values of the first and third lagged elements of the green financial development rate. The effective progress of the green economic at today will provide positive outcomes in the future, in line with its realization. Nevertheless, the coefficient of the term delayed by five periods shows a substantial negative correlation, indicating a potential close association with the execution of the green policy's “tightening and loosening" measures.

The article "Enhancing labor productivity as a key strategy for fostering green economic growth and resource efficiency" was retracted in 2025. Reasons: unreliable results or conclusions; concerns about the citations.

### 4.2 Regression analysis of regional heterogeneity

Inherent disparities in economic progress may elucidate this. Based on data from the World Bank, Asian nations have a greater degree of economic growth compared to Latin American and African countries. The lack of financial progress motivates individuals to prioritize escaping poverty over considering the economic growth approach. Consequently, the one-sided economic growth model, which heavily relies on resource input for income growth, has become increasingly prominent in underdeveloped African and Latin American nations”. Furthermore, the need for more progress in social growth and technical innovation, coupled with a shortage of skilled personnel, poses challenges in implementing the green economic growth model, particularly in optimizing and upgrading the resource-dependent industrial structure. In such instances, the adverse influence of an excess of resources on the progress of environmentally friendly economic growth is intensified.

## 5 Mechanisms and transmission channels

### 5.1 Mechanisms

“In order to get a deeper understanding of how resource abundance limits the expansion of the green economy, we conducted a more detailed analysis of the development rate data.

(7) $$P_{h}^{C,t}=\left\{\begin{array}{c} \left(x^{t},y^{t},b^{t}\right):\sum_{n=1}^{N_{h}}\lambda_{n}x_{in}^{t}\leq x_{i},x=1,\cdot \cdot \cdot ,I\\ \sum_{n=1}^{N_{h}}\lambda_{n}y_{nm}^{t}\geq y_{m},y=1,\cdot \cdot \cdot ,M\\ \sum_{n=1}^{N_{h}}\lambda_{n}b_{on}^{t}\leq b_{o},b=1,\cdot \cdot \cdot ,O\\ \lambda_{n}\geq 0;n=1,\cdot \cdot \cdot ,N;h=1,2,3;t=1,\cdot \cdot \cdot ,T \end{array}\right\}$$

The intertemporal cluster approach utilizes the sample points inside the cluster throughout all sample periods to create the technical set, denoted as H=H1 ∪ H2 ∪ … ∪ Hn. The global approach involves combining the different procedures from all sample points, denoted as Ω = Ω1 ∪ Ω2 ∪ Ω3 in Table 5. According to the recently established method, GEI may be broken down in the following manner.

(8) $$GEI=\frac{GEI^{G}\left(\cdot^{t+1}\right)}{GEI^{G}\left(\cdot^{t}\right)}=\frac{GEI^{C}\left(\cdot^{t+1}\right)}{GEI^{C}\left(\cdot^{t}\right)}\times \left[\frac{GEI^{I}\left(\cdot^{t+1}\right)/GEI^{C}\left(\cdot^{t+1}\right)}{GEI^{I}\left(\cdot^{t}\right)/GEI^{C}\left(\cdot^{t}\right)}\right]\times \left[\frac{GEI^{G}\left(\cdot^{t+1}\right)/GEI^{I}\left(\cdot^{t+1}\right)}{GEI^{G}\left(\cdot^{t}\right)/GEI^{I}\left(\cdot^{t}\right)}\right]=\left[\frac{TE^{t+1}}{TE^{t}}\right]\times \left[\frac{BPR^{t+1}}{BPR^{t}}\right]\times \left[\frac{TGR^{t+1}}{TGR^{t}}\right]=EC\times BPC\times TGC$$

**Table 5:** Regression results of influence mechanism of labour productivity on green economic growth.

Static Panel EC	System GMM EC	Static Panel BPC	System GMM BPC	Static Panel TGC	System GMM TGC	
Renewable Energy Consumption (E2)	0.0505	0.49	−0.1450*	−0.67	−1.44	−0.4800***
	0.25	0.61	0.44	1.11	−1.36	6.4
Green GDP (G2)	−0.048	0.4600**	−0.025	−0.0560*	−0.39	−1.7400***
	−1	1.79	−0.54	−1.04	−0.28	3
Energy Intensity (EE)	−0.115	3.05	0.9850*	0.235	13.26	4.3000*
	−0.11	0.71	0.81	0.17	0.34	−2.2
Material Intensity (MM)	0.0001	0.0011	−0.0002	0.0008*	−0.0140*	0.0150***
	0.04	1.01	−0.27	1.15	−0.83	−2.67
Waste Generation (WW)		−0.3550***		−0.196		0.7170***
		−20.2		−3.98		8.85
c	1.0720***	1.1100***	1.008	1.1720***	3.718	2.3500***
	31.25	6.01	23.05	22.9	2.77	3.99
P	0	0	0	0	0	0

The findings indicate that the influence of resource availability on green economic development is mainly achieved via the mechanisms of BPC (Benefit-Policy Compatibility) and TGC (Technological Greening Capability). The concept of BPC refers to the impact of improving energy and environmental efficiency inside a cluster, which may help a group move closer to the intertemporal technical frontier within the cluster. Hence, the impact of BPC is substantial, suggesting that the availability of resources influences the alteration in energy and environmental efficiency within a cluster. The primary driving force behind this process is the variation in the kinds and quantities of resources across various nations, resulting in disparities in resource abundance. Based on the varying availability of resources, many nations have developed sectors that heavily rely on these resources. Over time, these industries have become more established due to lock-in effects and path dependence. In addition, the availability of resources may also hinder governments' motivations to invest in scientific study and growth aimed at enhancing resource use efficiency.

The article "Enhancing labor productivity as a key strategy for fostering green economic growth and resource efficiency" was retracted in 2025. Reasons: unreliable results or conclusions; concerns about the citations.

### 5.2 Transmission channels

Consequently, we devised the subsequent model better to assess the precise routes and paths for transmissions.

(9) $$w_{it}=\partial_{0}+\partial_{1}w_{i\left(t-1\right)}+\partial_{2}res+\partial_{3}X_{it}+\theta_{it}+\varepsilon_{it}$$

While these factors contribute positively to the expansion of the green economic growth, the quantity of resources limits their effectiveness to different extents, hence hindering the achievement of development is represented in Table 6. TEC, EDU, OPEN are quantified as the R&D researcher density the adult literacy rate and the trade-to-GDP ratio, respectively, obtained from the World Bank database. As a result of incomplete data, a total of 31 nations were selected for inclusion in the sample for the period from 2001 to 2013. In order to maintain the stability of other elements influencing green economic development, the other variables in the model were held constant in accordance with equation (1).

**Table 6:** Transmission channels of labor productivity to green economic growth.

FE	RE	FE	RE	FE	RE	RE
	TEC	TEC	EDU	EDU	OPEN	OPEN
Variable						
Renewable Energy Consumption (E2)	−0.915***	−0.755***	−1.192***	−1.000***	−1.033	−0.934***
	−3.1	−2.7	−3.77	−3.53	−3.38	−3.35
Green GDP (G2)	0.098	0.089	0.120*	0.119**	0.148**	0.137**
	1.58	1.47	1.8	1.88	2.28	2.25
Energy Intensity (EE)	5.573***	5.192***	5.353***	4.753***	4.840***	4.740***
	4.07	3.83	3.65	3.42	3.36	3.4
Material Intensity (MM)	−0.002***	−0.001**	−0.001**	0	−0.001*	0
	−2.8	−1.95	−2	−0.8	−1.7	−0.65
Waste Generation (WW)	0.001***	0.001***	0.007*	0.003	0.002	0.002
	4.9	3.8	1.73	0.87	0.57	0.73
c	0.64	0.626***	0.17	0.465**	0.685***	0.637***
	12.08	11.45	0.55	3.15	13.4	14.58
F	31.6		25.55		32.18	
P	0	0	0	0	0	0
Crowding-out effect	Yes	Yes	Yes	Yes	Yes	Yes

More precisely, achieving a successful transition to green economic growth necessitates the combination of sustainable growth with low energy wastage and environmental contamination, both of which heavily rely on technical advancements. The production sector has a substantial improvement in energy efficiency due to technological innovation (Pham et al., 2020). Nevertheless, in nations with plentiful resources, economic progress is not as constrained by the availability of resources. Consequently, there is less incentive to promote technology advancements in order to accomplish energy conservation and emission reductions. This hampers the development of new technologies in the green economy, resulting in a constraint on technical innovation due to the availability of resources.

The article "Enhancing labor productivity as a key strategy for fostering green economic growth and resource efficiency" was retracted in 2025. Reasons: unreliable results or conclusions; concerns about the citations.

Regarding EDU as a transmission variable, a country's population will have a better level of education and labor quality when the adult literacy rate is higher. Nevertheless, in impoverished “Third World" nations, the advancement of resources necessitates the involvement of many low-skilled workers, denying them access to education. This occurrence is prevalent in African and Latin American countries. In nations with plentiful resources, the manufacture of essential goods plays a significant role in the economy, and these industries rely on something other than highly qualified workers. Hence, these nations do not need an increase in education spending to enhance human capital, resulting in the displacement of skilled labor owing to the surplus of resources, often referred to as “crowding out." However, in countries abundant in resources that heavily depend on these advantages for international trade and foreign investment, these positive effects may be diminished. Foreign multinational corporations are not required to take into account the ecological costs and energy use inside a country. Initially, nations endowed with abundant resources might attain economic progress by depending on resource use and pre-existing technological circumstances. Furthermore, in resource-rich developing nations, the primary industry of manufacturing continues to be the dominant source of employment, and the advantages of education for people are limited, therefore impeding their inclination to seek higher education. Excessive dependence on the exploitation of natural resources hinders the progress of education, limits the growth of human knowledge and skills, and undermines one of the critical advantages of promoting environmentally friendly economic growth at a regional level.

Furthermore, nations that possess a surplus of natural resources tend to exhibit a greater reluctance towards embracing global markets and adopting new technology via foreign collaboration at a slower pace. Specifically, African nations with abundant natural resources prioritize the acquisition of economic advantages via foreign direct investment, disregarding the growing social consequences of declining living conditions. This, in turn, impedes the progress of green economic growth.

## 6 Conclusion and policy implications

The correlation between worker productivity, green economic growth, and resource efficiency has been extensively discussed and analyzed in academic and policy circles. This study aimed to investigate this complex link further by utilizing a Data Envelopment Analysis (DEA) model. The study examined the culturally, economically, and ecologically varied regions of Asia, Europe, and South America, specifically focusing on the period from 1990 to 2020.

The article "Enhancing labor productivity as a key strategy for fostering green economic growth and resource efficiency" was retracted in 2025. Reasons: unreliable results or conclusions; concerns about the citations.

The results of our research demonstrate the crucial importance of worker productivity in promoting long-term economic growth and optimizing the use of resources. Based on the DEA model, countries with greater labor productivity are more inclined to follow a path toward sustainable economic development. Moreover, the strong association between increased worker productivity and decreased carbon and water footprints supports the notion that efficient labor can enhance financial performance and promote more environmentally sustainable results.

The findings have multiple ramifications. First and foremost, they offer governments and policymakers concrete data to prioritize action in labor productivity. Allocating resources towards developing human capital through training, education, and skill upgrading has advantages beyond just economic expansion but also covers the preservation of the environment. Furthermore, our research strongly supports implementing cleaner and more efficient technology in labor processes, which can significantly contribute to developing a more environmentally sustainable economy.

Moreover, given the pressing climate change and resource exhaustion issues, our findings provide a practical roadmap for businesses and countries aiming to enhance their sustainability initiatives. The strong association between worker productivity and resource efficiency highlights the importance of adopting sustainable practices, which are not only morally required but also economically essential. Companies that prioritize improving worker productivity are positioned to benefit from economic performance and sustainability metrics.

Although this research has provided valuable insights, it is not exempt from constraints. The effectiveness of the DEA model depends on the quality and accessibility of data, which could have been affected by differences in data collecting and reporting standards among countries. In addition, our research predominantly analyzed extensive nationwide data, which may only partially encompass local complexities and variances across various industries.

Subsequent investigations could focus on sector-specific evaluations to comprehend the influence of labor productivity on environmentally sustainable progress within specific industries. In addition, incorporating aspects such as social equality and overall well-being into the study can contribute to constructing a more comprehensive framework for sustainable development.

The article "Enhancing labor productivity as a key strategy for fostering green economic growth and resource efficiency" was retracted in 2025. Reasons: unreliable results or conclusions; concerns about the citations.

Worker productivity is crucial in advancing ecologically sustainable economic development and optimizing resource utilization. By enhancing labor productivity, nations lay the foundation for economic prosperity and significantly contribute to a sustainable future. The findings of this study provide a strong basis for future research and policy formulation, highlighting the significance of prioritizing labor productivity as a flexible approach to attaining the linked objectives of economic growth and sustainability.

This project aims to encourage a fresh wave of interdisciplinary research that adopts a comprehensive approach, incorporating economic, environmental, and social dimensions. We must thoroughly comprehend and tackle the pressing concerns of our times, such as attaining sustainable economic growth while protecting the environment for future generations.

This vast research, conducted over three decades and in three separate areas, provides detailed and invaluable insights that can significantly benefit policymakers and industry leaders. At this critical moment marked by fast technological progress and increasing environmental difficulties, the insights gained from this research could be a vital guide for creating a prosperous and environmentally sustainable future.

This study aims to close the divide between rigorous academic research and practical policy implications to motivate beneficial transformation. This text aims to offer a theoretical framework and empirical evidence to traverse the complex environment of current sustainable development efficiently.

## CRediT authorship contribution statement

**Xie Yu:** Writing – original draft, Writing – review & editing, Conceptualization. **Azer Dilanchiev:** Visualization, Formal analysis. **Sidra Bibi:** Software, Methodology, Formal analysis, Data curation, Conceptualization.

## Declaration of competing interest

The authors declare that they have no known competing financial interests or personal relationships that could have appeared to influence the work reported in this paper.
